The article "Development and Characterization of a Nanobody against Human T-Cell Immunoglobulin and Mucin-3" was retracted in 2023. Reasons: signs of a paper mill; suspected computer-generated content; unreliable results or conclusions; concerns about the data.

# Development and Characterization of a Nanobody against Human T-Cell Immunoglobulin and Mucin-3

**DOI:** 10.1155/2022/2929605

**Published:** 2022-06-11

**Authors:** Mingyuan Xia, Xiangnan Hu, Qiuxiang Zhao, Yi Ru, He Wang, Fang Zheng

**Affiliations:** ^1^Department of Urology, The Second Affiliated Hospital of Air Force Military Medical University, Xi'an City, 710032 Shaanxi Province, China; ^2^No. 986 Hospital, Air Force Military Medical University, Xi'an City, 710054 Shaanxi Province, China; ^3^Department of Biochemistry and Molecular Biology, Basic Medical College, Air Force Military Medical University, Xi'an City, 710032 Shaanxi Province, China; ^4^The Key Laboratory of Environment and Genes Related to Disease of Ministry of Education, Health Science Center, Xi'an Jiaotong University, Xi'an 710049, China

## Abstract

Monoclonal antibodies and antibody-derived biologics are essential tools for cancer research and therapy. The development of monoclonal antibody treatments for successful tumor-targeted therapies took several decades. A nanobody constructed by molecular engineering of heavy-chain-only antibody, which is unique in camel or alpaca, is a burgeoning tools of diagnostic and therapeutic in clinic. In this study, we immunized a 4-year-old female alpaca with TIM-3 antigen. Then, a VHH phage was synthesized from the transcriptome of its B cells by nested PCR as an intermediate library; the library selection for Tim-3 antigen is carried out in three rounds of translation. The most reactive colonies were selected by periplasmic extract monoclonal ELISA. The nanobody was immobilized by metal affinity chromatography (IMAC) purification with the use of a Ni-NTA column, SDS-PAGE, and Western blotting. Finally, the affinity of TIM3-specific nanobody was determined by ELISA. As results, specific 15 kD bands representing nanomaterials were observed on the gel and confirmed by Western blotting. The nanobody showed obvious specific immune response to Tim-3 and had high binding affinity. We have successfully prepared a functional anti-human Tim-3 nanobody with high affinity in vitro.

## 1. Introduction

Tumer immunotherapy with blocking immune checkpoint receptors as the core is considered as a pillar of cancer treatment for its advantages on security and potency. With the clinical validation of Ipilimumab and nivolumab (targeting checkpoint CTLA-4 and PD-1, respectively) [1], emerging checkpoints like mucin-domain-containing molecule-3 (TIM-3) and T-cell immunoglobulin have been identified sequentially. Belonging to the TIM family, TIM-3 is expressed on the cell envelope and functions as an immunoregulation receptor [2]. These proteins possess a common structure comprising an amino-terminal immunoglobulin variable domain with 5 noncanomical cysteines, and one each of mucin stalk, transmembrane domain, and cytoplasmic tail [2]. TIM3 was first identified as a membrane protein on Th1 cells, regulating macrophage activation [3]. In subsequent studies, it is found that TIM-3 is expressed in many other cellular types including CD4^+^ and CD8^+^ T cells, regulatory T lymphocytes, myeloid cells, natural killer cells, and mastocytes [3–7].

The article "Development and Characterization of a Nanobody against Human T-Cell Immunoglobulin and Mucin-3" was retracted in 2023. Reasons: signs of a paper mill; suspected computer-generated content; unreliable results or conclusions; concerns about the data.

TIM-3 ligands include galectin-9, high-mobility group box 1, and phosphatidylserine, as well as carcinoembryonic antigen-related cell adhesion molecule 1(CEACAM-1), the newly discovered one. It has been demonstrated in a variety of disease models that TIM3-galectin9 interaction suppresses immune responses [8–11]. Blocking of TIM-3 has been shown to increase quantity and IFN-*γ* secreting of CD4^+^T cells [12]. Numerous studies have shown that TIM-3 is positively correlated with tumour immune escape [13, 14], and the exhaustion of CD8^+^ T cells in models of chronic infection and tumours can be reactivated by antibodies against TIM-3 [14, 15].

Compared with programmed death receptor 1(PD-1) and cytotoxic T lymphocyte associated-4 (CTLA-4), two classic checkpoint receptors, the feature of TIM-3 lacks known inhibitory signaling motifs in its cytoplasmic tail [16], which suggests different mechanism of receptor action between TIM3 and classic checkpoints. This makes TIM-3 an excellent costimulation target for checkpoints containing immunoreceptor tyrosine based switch motif (ITSM) or immunoreceptor tyrosin-based inhibitory motif (ITIM). Furthermore, TIM-3 is mainly expressed in tumor infiltrating lymphocytes (TILs) [4, 5]. Thus, it reduces the damage to normal tissues when it is used as an immunotherapy target. So far, a variety of antibody formulations targeting TIM3 have entered clinical trials phase I/II, including monotherapy and coblocking with lymphocyte activation gene 3 (LAG-3) or PD-1 [17].

Nanobody constructed by molecular engineering of heavy-chain-only antibody, which is unique in camel or alpaca, is a burgeoning tools of diagnostic and therapeutic in clinic. Various advantageous properties of nanobody like decreased immunogenicity, high affinity, favorable dissolvability, and stability, binding to hinder epitopes and high yield expression in Escherichia coli or yeast result from their structure which contains only the heavy-chain variable domain of the heavy-chain-only antibody (VHH) [18]. Therefore, a variety of nanobodies targeting checkpoint receptors have been developed and reported while nanobody against TIM3 was reported twice by Homayouni et al. in 2016 [19] and Zhu et al. in 2018 [20], respectively.

The article "Development and Characterization of a Nanobody against Human T-Cell Immunoglobulin and Mucin-3" was retracted in 2023. Reasons: signs of a paper mill; suspected computer-generated content; unreliable results or conclusions; concerns about the data.

However, detailed evaluation of affinity and biological effect of TIM-3 specific nanobody is still lacking so far. The novelty and main purpose of this study is to evaluate the affinity and biological effect of TIM-3 specific nanobody constructed by molecular engineering of heavy-chain-only antibody, which is unique in camel or alpaca. Hence, in the present study, we developed and characterized TIM-3-specific nanobodies starting from alpaca immunization, purified and evaluated multiple indicators of them, and tested their ability of immune activation.

## 2. Materials and Methods

### 2.1. Alpaca Immunization and Effect Evaluation

A 4-year-old female alpaca introduced from China was subcutaneously injected with 100 *μ*g purified human TIM-3 protein (Sino Biological, Inc.) plus adjuvant FAMA (Gerbu, Germany) once a week. Peripheral blood was collected from jugular vein before the first injection and 7 days after the last injection, and serum was isolated by Sepmate tubes for comparison of the antibody titer by ELISA. A 96-well microplate well (Nunc, Danmark) was coated with 100 *μ*L 1 *μ*g/mL TIM-3 protein, and blank wells were coated with PBS. After washing and blocking, the preimmunization and postimmunization serum was added at serial dilutions. HRP-conjugated goat against Llama antibody (Thermo) was added as the II antibody, followed by the addition of ABTS reagent for the development of reaction. The measurement of OD (405 nm) was performed with the use of a microplate reader (Bio-Rad). All animal experiments were carried out with the approval of the relevant ethics committee and in strict accordance with the relevant regulations on the care and use of experimental animals in the international code of ethics and national health guidelines.

### 2.2. Library Construction

Using Sepmate tubes (STEMCELL) and Lymphoprep (STEMCELL), 100 mL peripheral blood was drawn to isolate peripheral blood mononuclear cells (PBMCs) 7 days after the last immunization. Trizol (Invitrogen)-separated total RNA from PBMCs was subjected to cDNA synthesis by SuperScript II reverse transcriptase (TAKARA) using random 6 primer. Then, via nested PCR, VHH gene amplification was done using primers CALL001 (5′-GTCCTGGCTGCTCTT CTACAAGG-3′) and CALL002 (5′-GGTACGTGCTGTTGAACTGTTCC-3′). The heavy chain antibody fragments (700 bp) were subjected to agarose gel (1%) electrophoresis and extraction via Quick Gel Extraction (Thermo) and then used as the template for the second PCR via primer VHH-sense (5′-CTAGTGCGGCCGCTGGAGACGGTGACCTGGGT-3′) and VHH-antisense (5′-GATGTGCAGCTGCAGGAGTCTGGRGGAGG-3′). These primers, designed for framework regions 1 and 4, involved restriction sites Pst 1 and Eco91I. The second PCR product was electrophoresed and purified by PCR Purification Combo Kit (Thermo). The phagemid vector pMES4 was digested with Pst 1, XbaI, and Eco91I restriction enzyme, while purified PCR product was digested with Pst 1 and Eco91I. The triple-digested pMES4 and double-digested PCR product was ligased with T4 DNA ligase enzyme (Invitrogen). After transfecting with the recombinant vector, chemically competent *E. coli* TG1 cells were subcultured on ampicilin-containing LB agar plates. Twenty colonies were randomly picked, and colony PCR was perform by vector primers GIII (5′-CCACAGACAGCCCTCATAG-3′) and MP57 (5′-TTATGCTTCCGGCTCGTATG-3′) to ensure that VHH was inserted into most of the transformants.

The article "Development and Characterization of a Nanobody against Human T-Cell Immunoglobulin and Mucin-3" was retracted in 2023. Reasons: signs of a paper mill; suspected computer-generated content; unreliable results or conclusions; concerns about the data.

Following infection of transformed TG1 with M13K07 helper phage (Invitrogen), the VHH library was displayed on phage. Infected bacteria were cultured overnight in 2× TY medium comprising ampicillin (AMP; 100 *μ*g/mL) and kanamycin (50 *μ*g/mL) while shaking (200 rpm). The medium was centrifuged for 15 min at 3200 g in 4°C. The supernatant was mixed with 20% ice cold PEG6000/NaCl and incubated for 30 min on ice. After centrifuged for 10 min at 3200 g in 4°C, such resuspended the phage pellet in ice cold PBS for biopanning.

### 2.3. Nanobody Library Biopanning

Three rounds of biopanning were performed on microplate wells coated with 100 *μ*L 1 *μ*g/mL TIM-3 protein in PBS to screen anti-TIM-3 phage displaying nanobodies. After blocking with 5% milk in PBS and 5 PBST rinses (250 *μ*L; 0.05% (*V*/*V*) Tween 20 in PBS), over 10^11^ p.f.u phage library preincubated in 0.1% milk in PBS was added into both well coated with TIM3 protein and PBS. Wells were washed with PBST for 15 times and eluted by adding 100 *μ*L 0.25 mg/mL trypsin solution per well for 30 min. The eluted phage was transferred into 100 *μ*L 10%BSA-PBS to stop protease reaction. The infecting log phase *E. coli* TG1 cells were obtained by serial dilution of 10 *μ*L phage eluted from wells coated with TIM-3 and PBS. 5 *μ*L drops of TG1 infected by dilutions of phage were pipetted on LB agar plate comprising AMP. The enrichment of phages carrying TIM-3-specific VHHs was identified by comparing the titers between phages eluted from antigen-coated wells and those from PBS wells. The rest of the eluted phages were applied to infecting log phage *E. coli* TG1 and cultured overnight to amplificate phage library as mentioned above for next round of biopanning.

### 2.4. Screening by Periplasmic Extract Monoclonal ELISA

*E. coli* TG1 cells infected by second and third round of phage sublibrary were subjected to overnight cultivation (37°C) on AMP-containing LB agar plates. 66 colonies from second rounds and 132 colonies from third-round sublibrary were picked randomly and cultured in TB medium containing AMP at 200 rpm in 37°C. Log phase *E. coli* TG1 were induced with 1 mM IPTG (Thermo) overnight (28°C). Via osmotic shock, the periplasmic proteins were extracted for ELISA using anti-HIS antibody (1 : 1000, Thermo), following by HRP-conjugated anti-mouse antibody(1 : 2000, Thermo) and TMB reagent. Anti-TIM3 (1 : 1000, Cell Signaling Technology) and HRP-conjugated anti-rabbit (1 : 2000, Cell Signaling Technology) antibodies were also added successively as the positive control. Positive clones were indicated if the OD450 in antigen-coated wells was three times higher than OD450 in PBS-coated wells. Clones considered positive were chosen for fragment sequencing and were classified according to CDR3 region.

The article "Development and Characterization of a Nanobody against Human T-Cell Immunoglobulin and Mucin-3" was retracted in 2023. Reasons: signs of a paper mill; suspected computer-generated content; unreliable results or conclusions; concerns about the data.

### 2.5. Nanobody Production and Purification

The TIM3-specific nanobody gene sequence was inserted into pHEN6c plasmid and transfected into *E. coli* WK6. His-tagged recombinant nanobodies were expressed in 1 L TB medium through 1 mM IPTG inducement and extracted via osmotic shock, followed by immobilized metal affinity chromatography (IMAC) purification with the use of a Ni-NTA column. The buffer of nanobody was exchanged from imidazole elution buffer to PBS by dialyzing.

### 2.6. SDS-PAGE and Western Blotting

Measurements of nanobody expression and purity were made by Coomassie brilliant blue stained 4%-20% SDS-PAGE and Western blot. The nitrocellulose membranes were transferred and blocked with 5% milk in TBST, and detected using anti-HIS (1 : 1000, Cell Signaling Technology) and HRP-conjugated anti-mouse (1 : 2000, Cell Signaling Technology) antibodies.

### 2.7. Affinity Measurement

Affinity of TIM3-specific nanobody was firstly determined by ELISA. Briefly, a 96-well plate coated by TIM3 protein or PBS overnight in 4°C and blocked with 5% milk PBS. A serial 10-fold dilution of nanobodies in 0.1% milk PBS was added. Antibodies anti-HIS (1 : 1000, Cell Signaling Technology) and HRP-conjugated anti-mouse (1 : 2000, Cell Signaling Technology) as well as TMB reagent were added into wells after washing, successively. The OD450 was measured, and the combination curve was drawn by GraphPad prism.

### 2.8. Statistical Processing

All statistical analysis was performed with SPSS 23.0 software (SPSS Inc., Chicago, IL, USA). All data are reported as the mean ± standard deviation (SD). Paired *t* test was used to compare the results in two matched groups. One-way ANOVA were applied to compare the differences between groups. *P* < 0.05 was considered as statistically significant.

The article "Development and Characterization of a Nanobody against Human T-Cell Immunoglobulin and Mucin-3" was retracted in 2023. Reasons: signs of a paper mill; suspected computer-generated content; unreliable results or conclusions; concerns about the data.

## 3. Results

### 3.1. Phage Display Nanobody Library Construction and Enrichment

After seven rounds of immunizations, the level of anti-TIM-3 antibody in alpaca serum was significantly increased as detected by ELISA (Figure 1(a)). The titer of specific antibody (both conventional heavy-chain-only antibody) after immunization appeared nearly two times higher than which was unimmunized until diluted to 10^5^. It demonstrated that one injection at weekly interval was sufficient to activate immune response of alpaca. Total mRNA from peripheral blood mononuclear cells (PBMCs) was isolated and was used as template to generate cDNA by RT-PCR. To prepare high purity VHH fragment library, nest PCR was used. The fragments of conventional antibody (1000 bp) and heavy-chain-only antibody (750 bp) were amplified simultaneously (Figure 1(b)) in first PCR. The primers annealing at framework 1 and 4, respectively, were made use of in second PCR, and 400 bp VHH fragments were amplified (Figure 1(c)). The PCR product, purified and digested, was ligated into phagemid vector pMES4 and transfected into *E. coli* TG1. The VHH library with a size of 3.7 × 10^8^ clones. PCR screening of 20 randomly picked colonies showed VHH inserts with proper size in most of the transformates (Figure 1(d)).

The VHH library was rescued by M13K07 helper phage and panned against recombinant TIM-3 protein coated in microplate wells. The enrichment of each rounds was monitored by titrate phage eluted from positive wells (coated with TIM-3 protein) and negative wells (coated with only PBS). After three rounds of panning, the enrichment ratio reached 3.8 × 10^3^ (Table 1), which suggest that it is sufficient to identify high affinity nanobodies.

Periplasmic protein was extracted from colonies infected by 2^nd^ and 3^rd^ round phage sublibrary, respectively. The periplasmic extract ELISA showed that 10 colonies represent significant binding that signal of their wells was three times higher than negative wells, of which R2G3 and R2C5 clone appeared even higher signal than commercial anti-TIM3 antibody. The rest of the nanobodies showed low-binding activity or poor expression (Figure 2). Positive clones were sequenced and classified according to complementarity determining regions, especially CDR3. Eight unique sequences containing the hallmark amino acid of nanobody are shown in Figure 3 (R3C1 is identical with R3B1 and R3E2 is identical with R3E1).

### 3.2. Production and Purification of TIM-3 Nanobodies

The fragment coding TIM-3-specific nanobodies was recloned into pHEN6c, the bacterial expression vector. Recombinant pHEN6c was then subjected to transformation into *E. coli* WK6. The generation of all nanobodies was completed in 1 L TB medium, and the purification was made via IMAC. The yield of nanobodies varied from 0.7 g to 14 g per liter. The washing buffer immidazol was changed by dialyzing to PBS. After verification of nanobody purity by Coomassie brilliant blue-stained SDS-PAGE (Figure 4(a)), Western blots were used to confirm expression and integrity of nanobodies (Figure 4(b)). It is demonstrated that all nanobodies were His tagged and located at 15 kDa on nitrocellulose membranes and gel.

The article "Development and Characterization of a Nanobody against Human T-Cell Immunoglobulin and Mucin-3" was retracted in 2023. Reasons: signs of a paper mill; suspected computer-generated content; unreliable results or conclusions; concerns about the data.

### 3.3. Affinity and Specificity of TIM-3 Nanobodies

We first determined affinity of nanobodies by ELISA. Serials of dilution of nanobodies were used to calculate Kaff values, based on which the mean affinity constants were generated. Primary affinity results are shown in Figure 5(a). Then, we tested the specificity of TIM-3 nanobodies by ELISA. A series of protein was used as negative control. It is shown that most of nanobody bound poorly with proteins expect for human TIM-3 (Figure 5(b)).

## 4. Discussion

The critical role of TIM-3 in immune cell exhaustion has been validated in multiple tumour and chronic infection models [21, 22]. T-cell immunoglobulin and Tim-3 are checkpoint receptors expressed by a wide variety of immune cells as well as leukemic stem cells [23]. TIM3 can be expressed on tumor cells and immune cells. It is expressed on a variety of immune cells, including Type 1 T helper cells (Th1), Th17 and CD8+ T cells, TILs, regulatory T cells (Tregs), and innate immune cells [24]. Depletion of T cells leads to T cell dysfunction in the immune response, preventing optimal tumor control. Conversely, in colorectal and prostate cancer, Tim-3 downregulation in tumor cells is considered a predictor of cancer progression [25, 26]. The proportion of TIM-3^+^ CD8^+^ T cells was detected to be notably increased in HIV-infected patients [27]. Blockade of TIM-3 with antibodies can recover TIM-3^+^CD8^+^ T cell proliferation. This phenomenon was found also in lymphocytic choriomeningitis virus infection, HBV infection, and some kinds of solid tumours, which makes TIM-3 an effective immunotherapy target. A study published in 2018 [28] suggests that blockade of PtdSer and CEACAM1 is a shared property of anti-Tim-3 antibodies with demonstrated functional efficacy. Now, Tim-3, one of several immune checkpoint suppressor molecules and one of the key mediators of cancer progression, has attracted attention as a target [29]. Kuang et al. [30] revealed a novel antibody targeting TIM-3 resulting in receptor internalization for cancer immunotherapy.

In this study, we successfully prepared a functional anti-human Tim-3 nanobody with high affinity in vitro. It is shown that anti-human Tim-3 nanobody obtains high affinity, which can be bound well with proteins. The affinity of different antibodies has been reported in the 10-7 to 10-10 m range [31]. Some studies have shown that very high affinity is suboptimal for therapeutic antibodies targeting solid tumors [19]. Since high-affinity antibodies tightly bind their specific antigens at the first contact, they will not go deep into the tumor around the tumor until all antigen molecules are saturated around the tumor [32]. However, there is still room for improvement; despite we have successfully prepared a functional anti-human Tim-3 nanobody, its functional effect and the diversity of the nanobodies' epitopes remains unknown. In the following research, we will determine the crystallographic structure of TIM-3 nanobodies to study the diversity of the nanobodies' epitopes. To delivering nanobody to malignant tissue sufficiently, a bispecific nanobody targeting both TIM-3 and prostate specific membrane antigen (PSMA) is being structured. The activity of bispecific nanobody will be tested by establishing a patient-derived tumor xenograft model using humanized immune reconstitution mice. The ability of bispecific nanobody in reactivation of TILs and restriction of tumour growth will be focused intensively.

The article "Development and Characterization of a Nanobody against Human T-Cell Immunoglobulin and Mucin-3" was retracted in 2023. Reasons: signs of a paper mill; suspected computer-generated content; unreliable results or conclusions; concerns about the data.

## Figures and Tables

**Figure 1:** Phage display nanobody library construction. (a) Evaluation of immunization effect by ELISA. Wells were coated with either 1 *μ*g/mL TIM-3 recombination protein or PBS. Serum before the first immunization and after the last immunization were detected by HRP-conjugated goat against Llama antibody and ABTS reagent. (b) The first PCR production had evident bands on 1000 bp and 750 bp. Lanes 1-4 represent different cDNA template quantities. (c) The 400 bp VHH fragments were amplified in second PCR. (d) 20 colonies were randomly picked and detected by PCR to calculate ratio of insert (18 positive colonies in 20.90%). ^∗^*P* < 0.05, compared to preimmunization.

**Figure 2:** Periplamic extract monoclonal ELISA (PE-ELISA) results of clones considered as positive. In total 10 clones expressed nanobodies react with TIM3 specifically. As is shown the R2G3 and R2C5 nanobody appeared higher signal than commercial TIM-3 antibody. The graph represents the mean of three experiments ± 3 SD.

**Figure 3:** Amino acid sequence of TIM-3 specific nanobodies. The frameworks and complementary determining regions were determined according to IMGT.

**Figure 4:** SDS-PAGE and Western blots to confirm purity and size of TIM-3 nanobodies (about 15 kDa). (a) 4%-20% SDS-PAGE shows nanobodies purified by immobilized metal affinity chromatography (IMAC). (b) Nanobodies were detected by anti-HIS antibody (1 : 1000) and HRP-conjugated anti-mouse antibody (1 : 2000).

The article "Development and Characterization of a Nanobody against Human T-Cell Immunoglobulin and Mucin-3" was retracted in 2023. Reasons: signs of a paper mill; suspected computer-generated content; unreliable results or conclusions; concerns about the data.

**Figure 5:** Affinity and specificity evaluation of TIM-3 nanobodies. (a) Serials of dilution nanobodies were tested on recombination using ELISA. R2G3 appears the highest binding capacity. (b) Nanobody R2G3 was tested on different coated protein using ELISA. c TIM-3 nanobodies epitope binning by SPR.

**Table 1:** Enrichment of phage after biopanning on TIM-3 antigen.

Rounds of biopanning	Input (pfu/mL)	Positive output (cfu/mL)	Negative output (cfu/mL)	Enrichment ratio	Output-input ratio
1	2.0 × 10^11^	7.0 × 10^6^	2.0 × 10^6^	3.5	3.5 × 10^−5^
2	1.1 × 10^12^	1.1 × 10^9^	7.0 × 10^6^	157.1	1.0 × 10^−3^
3	4.0 × 10^14^	8.0 × 10^9^	2.1 × 10^6^	3809.5	2.0 × 10^−5^

cfu: colony forming unit.

## Data Availability

The labeled dataset used to support the findings of this study are available from the corresponding author upon request.
